# Views of ophthalmologists on the genetics of age-related macular degeneration: Results of a qualitative study

**DOI:** 10.1371/journal.pone.0209328

**Published:** 2018-12-20

**Authors:** Julika Loss, Daniel Müller, Johannes Weigl, Horst Helbig, Caroline Brandl, Iris M. Heid, Robert P. Finger, Bernhard H. F. Weber, Janina Curbach

**Affiliations:** 1 Medical Sociology, Institute for Epidemiology and Preventive Medicine, University of Regensburg, Regensburg, Germany; 2 Department of Ophthalmology, University Hospital Regensburg, Regensburg, Germany; 3 Department of Genetic Epidemiology, University of Regensburg, Regensburg, Germany; 4 University Eye Hospital, University of Bonn, Bonn, Germany; 5 Institute of Human Genetics, University of Regensburg, Regensburg, Germany; University of Utah, UNITED STATES

## Abstract

**Background:**

Age-related macular degeneration (AMD) is the leading cause of blindness in industrialized countries. It is a multifactorial disease of the retina modified by environmental/individual (e.g. smoking) and genetic factors. 34 independent genomic loci are associated with the risk to develop AMD; an interaction between smoking and genetics is currently investigated. It is unclear how the knowledge on the strong genetic component has entered the knowledge base of practicing ophthalmologists, and how they inform and counsel their (AMD) patients about it. In this study, we explore the ophthalmologists’ view on AMD genetics, and their inclination towards communicating genetic risks to patients.

**Methods:**

We recruited a purposive sample of thirty German ophthalmologists (office based: n = 15, hospital employees: n = 15, f:8/30), who took part in a recorded semi-standardized interview. Transcripts were analyzed using content analysis.

**Results:**

The majority of office-based ophthalmologists claimed to be unfamiliar with genetics of AMD, in contrast to hospital-affiliated ophthalmologists. Both office and hospital ophthalmologists were convinced that genetics lacks practical relevance in everyday patient care. Many withhold information on heritability or genetic background of AMD from patients and their relatives, for fear of unsettling those individuals. The relevance of the genetic component of AMD or an individuals’ high genetic risk for prevention, e.g. screening or lifestyle modifications in persons with adverse genetic profile, was rated low.

**Conclusion:**

Developing genetic educational programs tailored to the routine care of ophthalmologists may be indicated, as well as a better two-way communication between research and practice. Exploring patient views about their expectations to being informed about genetic disease etiology, or about their individual risk, would help inform communication strategies.

## Introduction

Age-related macular degeneration (AMD) is the leading cause of blindness in industrialized countries. Its prevalence increases with age; in the population over the age of 65 years, 15–24% are affected by early stages of AMD, according to European population-based studies [1–3]. The prevalence can be expected to continue to rise as life expectancy is continuously increasing worldwide. AMD is differentiated into early or intermediate stages with drusen—amorphous extracellular deposits in the retina—and characteristic pigmentary changes, and late stages which may either be of the dry, atrophic type (geographic atrophy) or of the wet, neovascular type where the newly formed blood vessels lead to leakage and tissue destruction [4]. Early disease is often clinically asymptomatic. It progresses slowly, and only 10–20% of patients evolve to late AMD, of which two thirds have neovascular and one third atrophic AMD [5]. Late forms are characterized by irreversible loss of central vision. Treatment is currently available only for the neovascular type: intraocular injections with anti-VEGF are not curative, but can effectively reduce angiogenesis and vascular leakage [6, 7].

Multiple genetic and environmental risk factors have been found to be associated with early and/or late AMD. Whereas some lifestyle modifications are considered potentially useful in the prevention of AMD [8, 9], age and genetic factors convey the largest risk. Recent advances in genetic research have led to greatly increased understanding of the genetic underpinnings of AMD [10, 11]. Above all, since 2005, genome-wide association studies (GWAS) have contributed to our concepts of genetics in AMD by identifying numerous genetic variants, known as risk alleles or polymorphisms, associated with late AMD [12, 13]. Many of the AMD risk-alleles are related to genes involved in the alternative complement cascade, e.g. the *CFH* gene on chromosome 1 [9]. By now, 52 independent common and rare AMD gene variants at 34 chromosomal loci have been confirmed genome-wide, which collectively account for about half of the heritability of the disease [11]. A genetic risk score of an individual can capture the cumulative genetic risk that an individual has for developing a disease. For late AMD, the 10% individuals in the highest genetic risk score group have a 44-fold increased risk compared to those 10% in the lowest genetic risk score group [11, 14]. Thus, AMD has a particularly strong genetic component. Such a strong genetic component bares a peculiar feature: it can transfer from patients to their relatives.

For a practicing ophthalmologist, the evolving knowledge on the strong genetic background on AMD can be challenging in his or her daily practice. Clinical practice guidelines, e.g. from the British NICE, recommend to inform the patient about the causes of AMD [15]. However, these guidelines do not offer specific recommendations on whether and, if yes, *how* to communicate to an AMD patient that AMD etiology is largely genetic, that the patient will be likely to have the disease due to his or her genetic profile, and that this also transfers—to some extent—to the risk for relatives. In that sense, the ophthalmologists are left alone with emerging facts, and it is unclear what conclusions they draw without guidance on communication strategies.

Diagnosed AMD patients will, as evidence now stands, not benefit clinically from knowing their genetic AMD risk. Therefore, many authors advise against genetic testing for AMD, arguing that improved outcomes for genotyped patients have not yet been demonstrated in prospective clinical trials [16, 17]. Also the American Academy of Ophthalmology, in its guideline on macular degeneration, explicitly discourages eye physicians and patients from using genetic testing [18]. However, the patient’s genetic risk may be shared by offspring and siblings, who might or might not feel that they have a right to know about this precondition. Persons at high genetic risk might show high motivation to change their lifestyle when they are aware of this genetic risk. These individuals need to be counselled on early diagnosis and applicable prevention and treatment [19]. Some authors indeed point out that genotyping may be a potential tool for identifying individuals who may benefit from more intense monitoring and/or preventive strategies [8, 9, 20]. Potential preventive strategies could pertain to cigarette smoking, which has been shown to be an independent risk factor for AMD with a relative risk of 1.8 for current smokers versus never smokers [21, 22]. There is evidence suggesting that a healthy diet (i.e. rich in fruit, vegetables and fish) and vigorous physical activity may lower the odds for early AMD [9, 23, 24]. Studies also imply that there is an association between obesity and AMD [25, 26]. Genetic risk factors interact with lifestyle modifications: gene-environment interaction studies have shown that genetic susceptibility can be altered by modifiable factors; e.g. the susceptibility to advanced AMD associated with variants at the *CFH* gene locus was shown to be modified by body mass index or adherence to a Mediterranean diet [24, 27]. There is recent evidence that lifestyle factors such as smoking can induce epigenetic changes that modify gene expression [9, 28]; research in this field is currently developing.

Gene-environment interactions are complex and not fully understand, which may render preventive lifestyle counseling difficult [29]. In terms of monitoring, early detection (e.g. via digital color fundus photographs) might be beneficial for individuals with an elevated genetic risk of AMD, as it enables timely referrals resulting in a better prognosis due to prompt therapy once late AMD (in its wet form) has developed [30, 31].

Ophthalmologists may be approached by relatives of AMD patients asking for advice, because some patient brochures about AMD mention the genetic background of the disease. As commercial genetic testing which screens for a number of common AMD risk variants is currently available [9, 12, 14], eye physicians may even encounter a patient with AMD or a relative with a genetic test result and need to handle this situation [5]. There is little information about the way eye doctors manage and communicate the genetics of the diseases they treat as part of their routine practice [19]. Available recommendations for ocular genetic counseling refer to monogenetic eye disorders, e.g. retinitis pigmentosa [32], but not to complex disorders where multiple genes may interact with each other and with environmental factors over a life course to manifest (or not manifest) the disease. Current clinical practice guidelines do not help ophthalmologists decide whom to inform about the genetics of AMD, and in what detail, and to what purpose. In addition, we do not know if and how ophthalmologists keep abreast of the genetic research on AMD, and how accessible the results are to them.

With the novel evidence on AMD genetics, ophthalmologists are left alone with new options and/or responsibilities for counselling (or not counselling) their AMD patients and/or their relatives on genetics, and they may encounter new demands by patients who are well informed about or interested in AMD genetics. There is no gold standard yet that could guide ophthalmologists in these situations. Therefore, the actual counselling procedures may range from withholding all evidence, over mentioning a general knowledge of genetic risk factors for AMD or a possible individual genetic predisposition, to discussing a presented genetic code from commercial genetic testing with a healthy person, a patient, or a patient’s relative. So far, it is unclear how far the increasing amount of genomic discoveries relating to AMD is reflected in the routine ophthalmologic care. We therefore set out to better understand what impact the evolving knowledge on AMD genetics has on clinical ophthalmologic practice, i.e. counselling patients and relatives. We also postulate that the perspectives of ophthalmologists on genetics is linked to their knowledge of AMD genetics, and to the way they learn about the results of genetic research. Specifically, the study intends to explore:

1. how familiar ophthalmologists (private practitioners and hospital employees) are with the genetics of AMD,
2. how they assess the information on AMD genetics that is available to them,
3. how relevant they consider genetics in their daily practice to be,
4. which advantages/disadvantages they attribute to potential genetic tests for AMD, and
5. how they communicate genetic aspects to their AMD patients and/or the relatives of AMD patients.

To that aim, we conducted a qualitative study with ophthalmologists, which could reveal the perspective of eye doctors on the scientific genetic developments in macular degeneration.

## Methods

### Organizational setting

In Germany, about 80% of ophthalmologists work in their own private practice, whereas about 20% are employed by hospitals. AMD patients are usually seen by private practitioners, who refer them to an ophthalmologic center in a hospital (usually university hospital) if for example intravitreal anti-VEGF injections are indicated. Over the last decade, an increasing number of office-based practitioners has started to perform the injections themselves.

### Study design

We conducted a cross-sectional qualitative study with the aim to explore views of ophthalmologists from two sub-samples: ophthalmologists who run a private practice (n = 15) and ophthalmologists employed by hospitals (n = 15). Initially, the research design was restricted to interviewing private practitioners in Eastern Bavaria (Germany). But early on in the interviews, two participating eye doctors remarked independently from each other that informing AMD patients about genetics would be of more importance in the university hospital setting, where doctors may have closer links to genetic research. Therefore, it was decided to extend the study to also include a sample of hospital-affiliated ophthalmologists, which were recruited from university medical centers across Germany, to be able to contrast the views of both sub-samples with each other.

### Data collection

We performed semi-structured face-to-face interviews with 30 ophthalmologists. The interview guide covered different aspects of genetics of AMD and communication with patients suffering from AMD: the doctor’s information sources about genetics, familiarity with AMD genetics, perceived clinical relevance of genetics (in the present and the future), and patient education on genetics. The interview guide was pilot-tested with two office-based ophthalmologists. For the final version of the interview guide see Table 1.

**Table 1:** Interview guide.

A. General aspects of communication with patients:
1. What topics do you discuss with AMD patients on their first consultation?
2. What topics do you discuss with AMD patients during their routine care?
B. Familiarity with and information on genetics:
3. Do you feel familiar with genetic aspects of AMD?
- If no: could you explain why not?
4. How do you educate yourself on genetics?
5. In your opinion, how accessible and understandable is the current information on AMD genetics?
C. Relevance of genetics in the care of AMD
6. In your opinion, how do results of AMD genetics contribute to the prevention and care of the disease?
7. In your opinion, is there a need to better link genetic research and daily ophthalmological practice?
D. Discussing genetics with patients and/or relatives
8. Do you mention that AMD may have a genetic component?
- If yes: could you outline your practical approach?
- If no: could you explain why not?
9. How do you handle questions about genetics?
10. Do you think there is a potential value for family members of AMD patients?
E. (Future) value of genetic testing
11. How would you assess the potential of genetic testing in the future?
- prompts: identification of patients at risk, personalized treatment

The interviews took place at the respective doctor’s workplace and were conducted from January to October 2016 by either of two researchers (DM and JW, both male doctoral students). The researchers had been intensively trained in the conduct of semi-structured interviews and already had experiences in qualitative data collection. The interviews lasted 17–36 minutes; they were audio-taped, transcribed verbatim, and de-identified. In addition, field notes were taken.

### Recruitment and sample

Office-based ophthalmologists were recruited in various towns and communities of Eastern Bavaria (Germany), hospital-affiliated ophthalmologists were recruited from eleven German university medical centers. Among the ophthalmologists in private practice, we sought to recruit a diverse sample including doctors of both genders, with longer and shorter post-qualification experience, and from urban, suburban, or rural areas (purposive sampling). 25 invitations per mail, followed by phone calls, were made; 10 doctors refused to participate, due to lack of interest and/or time. To recruit hospital-affiliated ophthalmologists, e-mail inquiries were sent to 17 consultants working at ophthalmology departments in university medical centers. These ophthalmologists were chosen because a special focus on AMD or retinal diseases was evident (publications, research projects), and via snow ball recruitment. Two of those contacted did not reply to e-mails even after repeated requests.

All interviewed ophthalmologists had finished their training in ophthalmology at least 5 years (up to more than 30 years) before and treated AMD patients on a daily basis. 8/30 interview partners were female (3 in the private practice sub-sample, 5 in the hospital sub-sample).

### Data analysis

The interview transcripts were numbered chronologically (IP 01—IP 30) and classified according to the work place of the doctor (o = office ophthalmologists; h = hospital employees) before de-identification. A qualitative content analysis was performed [33], identifying thematically related sections across interviews. In order to ensure proper categorization of the data, the transcripts were repeatedly read before and after coding. Categories were initially developed based on the underlying interview guide, but in the analytic process, new topics emerged within each main category. Once established categories were repeatedly re-assessed and adapted to new aspects. In order to enhance the validity of the findings, the transcripts were read and coded independently by three authors (DM, JW and JL), differences in categorization were discussed until consensus was reached. Discrepancies in results, contradictory aspects and deviant statements were analyzed with particular attention [34]. All authors involved in the data analysis agreed that data saturation was reached in both sub samples, i.e. no more new themes appeared in the last interviews. The study reporting considers the criteria suggested in the COREQ checklist (consolidated criteria for reporting qualitative studies) [35].

### Informed consent and ethics approval

All procedures were in accordance with the ethical with the Helsinki Declaration of 1975, as revised in 2000. All participants gave their informed consent to be interviewed and recorded. In order to ensure confidentiality of information, only two researchers were involved in data collection and transcription. The transcripts were de-identified before analysis, so nobody except for the interviewer could link the statements to a certain ophthalmologist or institution. The study was approved by the ethical review committee of the University of Regensburg (Ref.-No.: 14-101-0237).

## Results

### Familiarity with AMD genetics and information seeking behavior

Among the 15 interviewed private practitioners, only one ophthalmologist claimed to feel well informed about AMD genetics (IP 01 o); the vast majority admitted not to be especially familiar with this issue. Their statements revealed differences in how detailed the knowledge of the interviewees was, ranging from a vaguely assumed heritability to explanations of specific gene variants.

*You know from the practice that there are simply families in which [AMD] seems to run. I’m not aware of the reason for this. I think this is not exactly known. …But to be honest, genetics is certainly an issue that I’m not well informed about*.

(*IP 05 o*)

*There are eight different genes, and if that and that many genes are positive, then the offspring will with a probability of x percent develop a macular degeneration when they’re old*.

(*IP 13 o*)

The interview partners who worked in their own private practice named different factors which prevented them from learning more about or understanding AMD genetics, mainly the dynamics and complexity of genetic research, as well as a general or relative lack of interest in the subject matter.

*[Genetic research] is currently in a state of flux […]. There’s a permanent change in what you can nail down genetically, and in this regard, it’s difficult*.

(*IP 10 o*)

*I stem from a generation of eye doctors, […] in which you knew that genetics exist, […] but basically, this wasn’t of any interest to us. And still today [genetics] is not my cup of tea*.

(*IP 05 o*)

Many private practitioners did not actively search for scientific information, but usually rely on being informed automatically in case of significant developments, using, as one interviewee put it, “*what the University delivers to my doorstep*” (IP 09 o).

*If there really is a big breakthrough, then I will get to know it anyway, by a CME course at the University or by a drug rep, because they need to sell this knowledge to the customers*.

(*IP07 o*)

In contrast, most of the ophthalmologists from university hospitals felt to be ‘up to date’ with the genetic research on AMD, mainly due to self-motivated literature searches or attended conferences. Personal contact to and research co-operations with genetic researchers also played a role.

*[I use] the Internet and papers, (…) but we also talk to colleagues from the Institute of Human Genetics here on a regular basis, as we work together in that field*.

(*IP 22 h*)

*[I get information about new research findings] at conferences or advanced training courses. Articles less so, because they are usually very specific and you have to do a lot of reading to get an idea of the content. That’s too time-consuming*.

(*IP 28 h*)

Some interview partners employed by hospitals reported that they had difficulties in keeping up with the progress in genetic research, e.g. due to time constraints or the vast amount of new publications.

*In the daily (…) struggle in the hospital, there’s much stuff that gets lost, and then you don’t have so much time to trawl all these papers [for genetics]*.

(*IP 16 h*)

*Genetics…by now, this has become very complex, so it’s not as easy anymore to get to the bottom of it (…). When you look into PubMed, (…) there are new things coming up every week, and I have a hard time sometimes to judge how relevant a new finding is—is it really something new, or is it just the same that had been published in 2005 and 2006?*.

(*IP 26 h*)

### Information sources and knowledge transfer

The above-mentioned information sources differed between private practitioners and hospital employees. Private practitioners mainly referred to German ophthalmological journals, some to textbooks, in which they mostly reported to come across articles on AMD genetics only once in a while. In contrast, hospital-affiliated ophthalmologists were more familiar with PubMed searches and international papers. Both groups also mention oral presentations, e.g. at CME events, as important information sources. The majority of those interview partners working in their own practice were not satisfied with the way the results were presented, especially in the journal articles, because these would lack simple, concise summaries and practical implications.

*It is rare to find articles about genetics…I do read those [articles], but for me, this is rather like advanced Latin. I take note of it, but I cannot keep that in mind to that extent*.

(*IP 06 o*)

*I have subscribed to different journals, which I sometimes read very intensively, sometimes less intensively. But about genetics of macular degeneration…? There’s basically nothing tangible in there …In most cases, it’s is so special that it overstretches the frame for practitioners*.

(*IP 05 o*).

Whereas hospital-affiliated ophthalmologists felt that an annual or biannual presentation of a geneticist would be sufficient to maintain an overview of significant developments in AMD genetics, the private practitioners stressed that those presentations would only be helpful if they were clear and referred to knowledge that can be utilized in their practice.

*[With oral talks] it is important that it’s not spaced out too much. If somehow one genome 533 is compared to genome 544, the normal eye doctor will not be interested*.

(*IP 14 o*)

### Clinical utility of genetics

With the exception of one hospital employee, who had specialized in genetic eye diseases and regularly performs genetic testing with his patients (IP 22 h), all ophthalmologists in both samples stressed that genetics did not play a role in the daily routine care of AMD patients. Genetic research and its results were described as ‘*virtual’* and ‘*divorced from reality’*.

*As far as genetics is concerned, this is partly in striking contrast to your everyday job—which is very much about mundane stuff. It is about whether the expenses for a walking stick are reimbursed, and not about whether some chromosome is somewhat crooked*.

(*IP 03 o*)

Different reasons were given for the limited clinical utility (see Table 2), especially a lack of therapeutic consequences.

**Table 2:** Reasons given for the limited clinical relevance of AMD genetics.

Reasons given for the limited clinical relevance of AMD genetics			
Categories	IP (n)*		Sample quotes
	office	hospital	
Inalterability of genes	2/15	0/15	*Practical relevance is missing*, *because nobody can take a pick of their genes*. *If they’ve got it*, *they‘ve got it*. *So I don’t even start trying to figure it out*, *because it doesn’t make sense*, *basically*. *(IP 07 o)*
Limited / unclear influence of genes on phenotype	4/15	0/15	*There are certainly some genes … in which the disease onset or the impairment in function differs between each gene carrier*. *(IP 06 o)* *What more can I say in terms of genetics*? *I mean*, *this is multifactorial and this is not as direct that it means that they really have to get [the disease]*, *isn’t it*? *(IP 10 o)*
Missing consequence for prevention	2/15	5/15	*[Genetics*:*] practical relevance for me is nil*. *Because the patient is* here, *and already has his or her problem*. *It [AMD] hasn’t been prevented*, *that you could have done anything to prevent it*. *That’s why genetics…doesn’t have any applicable use for me in the daily work*. *(IP 09 o)* *There is a high association between the development of AMD and genetic defects*, *but currently*, *it has not a single consequence in the daily clinical work*. *I can’t send a patient with AMD*, *or even prophylactically*, *to a human geneticist*. *What is the point of that*? *(…) It has little relevance and consequence*. *(IP 20 h)*
Missing consequence for therapy	6/15	6/15	*[The patient] probably doesn’t care which allele is altered on which gene*, *and they also don’t care what will be in 10 years’ time… but when they ask me today*: *‘Why is it that I can’t drive my car anymore*, *and why is it that there is no medication against it*?*’*, *then there’s nothing I can offer them*. *(IP 03 o)* *Currently*, *it is good to know [about genetics]*, *but there isn’t any consequence*. *Nothing changes with respect to the therapy or the progression of the disease*. *(IP 30 h)*
High age of patients / late stage of disease	2/15	1/15	*Most people who …suffer from macular degeneration are 70*,*75*, *80 years [old]*, *and the disease has progressed so far that I can’t imagine that there’s anything left to be done by genetics or gene therapy*. *(IP 12 o)* *If I told them about complement factor H and risk alleles*, *it wouldn’t be of any help for most of the patients*. *(…) Family planning is of no importance in that age group*. *(IP 25 h)*
Lack of interest from patients	0/15	1/15	*Because there is little feedback [from the patients]*, *…the genetic component … doesn’t play a role in the ordinary doctor’s consultation*. *(IP 22 h)*

*Please note that these were points that were brought up by the interview partners themselves when openly asked about reasons, or when being asked to explain the low relevance. Numbers may certainly have been higher if all these reasons had been explicitly asked for in an ‘agree’/‘disagree’ way.

### Knowledge exchange between research and practice

Some interviewed ophthalmologists pointed out that there is a gap between genetic research and practice, mainly due to a lack of communication between genetic scientists and ophthalmologists, leading to non-transparency. According to some office-based interview partners, genetic research results which cannot easily be translated into recommended actions in clinical practice run the risk of being irrelevant. In that sense, a better two-way communication was proposed.

*It takes scientists who know their way with genetics, and who push that issue forward. In order to translate this into clinical day-to-day practice—well, this is the missing link. It would be nice if there was something being developed for the future*.

(*IP18 h*)

*What is the geneticist doing? What? What? Are they trying a shot in the dark? What do they want? Why are they doing research? Do they have a clear direction? It may well be that this direction is completely contrary to ours*.

(*IP 13 o*)

*I would recommend, and this is an appeal to the universities, that they get in touch with the practitioners, that they approach us, not the other way around, and start a dialogue. This is desperately needed*.

(*IP 08 o*)

### Informing AMD patients about genetics of the disease

Some office-based ophthalmologists, and most of the hospital employees, report that they principally educate their AMD patients on the genetic background of their disease. Normally this education is only rather superficial, ‘*rather one sentence only*’ (IP 22 h), e.g. just mentioning that the macular degeneration can be hereditary, which is also attributed to time constraints.

*We don’t say something about special mutations… We say: ‘There may be a genetic component. There are hints that it can run in the family.’ That’s all we say about it*.

(*IP 19 h*)

Few interview partners explained that they only talked about genetics, or hereditability, when the patients ask about it. Some interview partners—from both settings—would principally avoid talking about AMD hereditability with their patients, as they saw no consequences, and because they did not want to unnecessarily burden or worry the patients with this knowledge.

*I don’t bring [genetics] up, deliberately. There are some patients which make the impression [that the disease runs in the family]. But this doesn’t matter… there’s one family, this is quite severe, where the daughter got [AMD] with fifty, and the mother with seventy. But it’s no use [talking about genetics]. The daughter has no children, won’t have any either. Why should I upset the apple cart?*.

(*IP 11 o*)

*You can’t change the genes anyway, so I don’t tell them [anything about genetic factors]. I can’t exactly say: ‘It’s your own fault! You’ve got a bad genetic profile!’. I don’t do that*.

(*IP 07 o*)

*[Genetics] has only little clinical relevance and possibly contributes to upsetting [patients] as well*.

(*IP 21 h*)

### Addressing relatives of patients with macular degeneration

Few interview partners ask their patients to inform their relatives about the genetic background of AMD and the possibility of ophthalmological screening.

*If a patient with macular degeneration has come to see me, I always mention that a certain hereditary component can play a role, and that maybe other family members should undergo a little medical check*.

(*IP 15 o*)

Many interview partners—in both samples—were reluctant, however, to address accompanying family members of their AMD patients and to point out a possible genetic component to them, or to recommend their patients to educate their relatives. The interview partners did not want to worry those relatives, especially because of the uncertain disease risk. When their patients explicitly ask about their descendants’ risk to get the disease, only some doctors would offer to see and screen those descendants; mostly they give very general information about hereditability and the difficult predictability of the disease.

*I don’t consider the risk of inheritance high enough to justify upsetting and unsettling a young person in a way that they go through their life, and with every visual phenomenon they have they believe that this is the outbreak of their macular degeneration right now*.

(*IP 21 h*).

*I’m not in favor of stirring up fears. Patients will notice early enough that something is wrong. And to burden them with worry for decades,—well there’s not enough evidence for that*.

(*IP 28 h*)

One interview partner also mentioned potential ethical problems in advising a person who is not one’s own patient.

*I don’t consider it my responsibility as a doctor to point out [the AMD risk] to an accompanying person, I even consider it almost ethically reprehensible. When we are asked directly, then of course we are answering that question, but in my opinion, this is also somewhat difficult when the question is asked by an accompanying person, who is basically not your patient*.

(*IP 27 h*)

The majority of office-based as well as hospital-affiliated ophthalmologists have already experienced being approached by family members of patients with macular degeneration (either as patients treated for other diseases, or as accompanying persons) and being asked about these persons’ individual risk to get the disease. The interviewed ophthalmologists have different strategies to deal with this request: The office-based ophthalmologists mostly screen the patients using fundoscopy, reassure the patients in case of a normal finding, and recommend regular check-ups every couple of years; some hand out Amsler grid cards, a simple device to self-test for distortions in a person’s vision. None of the interviewed ophthalmologists recommend genetic testing or calculating risk scores. Amongst the hospital employees only a few interview partners stated that they would give some further advice to the patients or their relatives in case of questions.

*The main focus is the patient, but (…) if the children are present, they often ask [about their risk]. Then I willingly tell them (…) that there is an inherent and an age-related component. And then actually I always recommend them to have their eyes examined*.

(*IP 23 h*)

### Genetic testing

One office-based ophthalmologist (IP 08 o) was convinced of the reliability of available genetic tests, and supported the use of these tests; all other interview partners were opposed to genetic testing. Among the office-based ophthalmologists, there were many interview partners who considered available genetic tests pre-mature or even dubious (“*marketing rubbish*”, IP 03 o); the predictive value was believed to be very low (“*not as relevant and conclusive*”, IP 01 o).

Beside this skepticism regarding the technical characteristics of genetic tests, the majority of interview partners—both office-based and hospital-affiliated—expressed the view that predicting the AMD risk genetically would not have any helpful preventive (or therapeutic, for that matter) consequences. The arguments for this view ranged from simple statements along the lines of “*you can’t change anything about it if someone has the genes*” (IP 06 o), to more sophisticated argumentations about preventive measures.

*If somebody has a completely normal vision, what’s in it for them if they have their genes checked? …with AMD, what are the consequences for this person, what’s their big advantage? You don’t know at all how the [trait] expression will be, and then an additional mental problem will be generated*.

(*IP 07 o*)

*Right now, we can’t derive a consequence from the [genetic] test (…). When you test a 20-year-old, and tell him or her: ‘Well, now we wait till you’re 60, and then we will start with the AMD prophylaxis’, then there is no need to test them with 20 in the first place*.

(*IP 25 h*)

*There are these genetic tests, but we don’t use or recommend it a big deal. On the contrary, we rather advise against it, because in the end, is has only little clinical relevance…What are you telling a patient you’ve identified? Well, you can tell him or her not to smoke… or you can point out the AREDS medication, although it isn’t clear yet whether this helps at all in this early stage*.

(*IP 21 h*)

Many interviewees were worried about the potential burden that the finding of a high genetic risk may pose upon a tested person. One interview partner also mentioned the possibility of a fatalistic reaction.

*In some cases, this means knowing, in one’s young years, ‘I’m a gene carrier’, and you mustn’t underestimate the fear that you’re imposing there … Okay, you can promote their awareness and their intention to live healthier. But you may as well chase somebody into the opposite direction … You mustn’t forget the patient’s psyche…Maybe you’re planting fears within somebody that are not required*.

(*IP 06 o*)

One interview partner pointed out that selecting patients who are entitled for gene tests would be challenging for doctors.

*How should I select? So there is some [patient] whom I grant the most sophisticated genetic testing in a high-end clinic… but why exactly this person? …I can’t test each potential AMD patient… but then, I would have to offer it to everybody, or to nobody. That’s where it starts to get a bit difficult*.

(*IP 03 o*)

None of the interviewees has ever experienced a patient or relative to bring up the topic of genetic tests themselves. When asked how they would react if a patient sought their advice on using a genetic test, the interview partners described different proceedings: some would clearly advise the patient against it, pointing out the uselessness of the test; some would accept if the patient wanted to undergo the testing, although trying to dampen their expectations; some would support a patient’s wish by enquiring local test options.

*I’d probably say: ‘If you absolutely want to do it, and to invest the money, then go ahead. But just don’t get your hopes up too high, and expect somebody to be able to tell you afterwards: ‘Now we’re going to do this and that, and then you won’t get macular degeneration.’ […]. I’d rather say: ‘It’s not worth it.’*.

(*IP 05 o*)

### Future potential of genetic research

Despite the predominantly negative attitude towards genetic testing, many interviewed ophthalmologists were confident about future benefits that genetic research would bring for AMD, especially in terms of personalized treatment. These perspectives, however, were rather vague.

*[Genetic tests]… in the long run, this will certainly be useful, and you will be able to do quite a lot of things, [e.g.] that, first thing, you check the whole thing genetically, and then treat the patient accordingly*.

(*IP 15 o*)

Some of the hospital- affiliated ophthalmologists had expectations that were better informed and more concise, especially with regard to personalized therapy of dry AMD.

*There are (…) first hints that patients with certain gene variants obviously react better to a medication, for example Lampalizumab, when treated for dry AMD, and possibly some sort personalized therapy will exist in the future. But for the time being, this is still a long way off*.

(*IP 20 h*)

## Discussion

### Main findings

The broad majority of office-based ophthalmologists claimed not to be familiar with genetics of AMD, mainly due to its complexity and dynamics; media such as German journals or CME lectures were reported not to bring about the results of genetic research in a comprehensive and meaningful way. The terminology used by many of the office-based ophthalmologists implies that they have not come to terms with the concept of multifactorial diseases yet; terms like ‘gene carrier’, or ‘in some patients, AMD seems to be genetic’ rather hint at the concept of monogenetic diseases. In contrast, hospital-affiliated ophthalmologists felt well-informed about the recent research developments in AMD genetics and gained knowledge not only by PubMed searches, but also through personal interaction with geneticists. Both groups were convinced that genetics has, for the time being, no practical relevance in everyday patient care; they felt that more practical utility could arise in the future if genetics helped personalize AMD therapy. The relevance of heritability or genetic testing for prevention, e.g. dense screening of those at high genetic risk for early diagnosis, or changing lifestyle with regard to risky behaviors, was rated low. Especially office-based ophthalmologists were struggling to link the concept of prevention to genetics and to the ophthalmologic care they provide to AMD patients, arguing that genes could not be changed or that primary prevention was not feasible anymore in patients with manifest AMD. Addressing relatives of AMD patients as persons with a higher genetic risk of AMD was dismissed by the majority of both office-based and hospital-affiliated ophthalmologists, mainly for ethical reasons (avoiding unnecessary burden as well as allocation and privacy problems). The doctors would even be reserved when directly asked by relatives about their risks. None of the interviewees has ever discussed (results of) genetic testing with their patients yet, the majority (but not all) would advise against it if directly consulted on this.

### Strengths and limitations

The number of 30 interview partners is small, so it cannot be assumed that the findings presented here are representative of the views of all ophthalmologists in Germany. However, the aim of qualitative studies is not to receive representative data, but to gain a deeper understanding of social and psychological processes and to capture the subjective views and experiences of the persons interviewed. Using a qualitative study design allowed us to tap personal attitudes and professional experiences of doctors that are not readily expressed in response to survey questions [33], and that are key to understand the complex processes and conditions involved in patient care. In addition, we strove to generate a balanced perspective by including both office-based and hospital-affiliated ophthalmologists, and by paying attention also to divergent attitudes. The use of only two interviewers for all participants (one for each subsample), and three independent researchers for data analysis ensured quality control and minimal interpretive bias.

### Comparison with other studies

The bulk of literature on medical doctors’ knowledge and training needs on genetics is focused on hereditary cancer, mostly breast cancer and colorectal cancer. Surveys among specialists in different countries revealed a lack of (perceived) knowledge and an ambivalent attitude towards genetic testing in cancer [36, 37], even though the genetics of breast and colorectal cancer are very present in the public (and scientific) discourse—much more than AMD genetics. Houwink et al [38] also performed a qualitative study exploring the role of genetics in patient care by conducting focus groups with Dutch general practitioners. Similar to our findings among office-based ophthalmologists, the Dutch general practitioners perceived deficiencies in their basic understanding of genetics, and they considered it difficult to access genetic information that is easy to understand and can be applied in daily practice. The Dutch sample also brought up a number of ethical dilemmas connected to genetic testing (disclosure, privacy), which corresponds well with the concerns of the ophthalmologists interviewed in our study. The main difference between the results of Houwink et al and our study was that the Dutch doctors expressed a clear and urgent need for better genetic education, as they experienced their lack of knowledge as a barrier in patient care; in our study, the majority of interviewed office-based ophthalmologists were reluctant to invest in learning about genetics, mainly because they felt that the topic was not clinically relevant. The difference may be explained by the fact that general practitioners, due to the wide range of conditions treated in primary care, may encounter diseases with a genetic background more often than ophthalmologists. In fact, the Dutch physicians reported an increase in patient inquiries about genetic issues, a phenomenon which is not reflected in the experiences of our sample of ophthalmologists. In addition, we asked about the relevance of genetics in a specific complex disease (AMD), whereas the Dutch study asked about genetics in general, also including monogenetic diseases. We are aware of only one study which has collected data among ophthalmologists on their perspective of genetics in eye diseases, a survey performed among 73 eye doctors in Brazil [19]. The study was probably conducted before the first GWAS results on AMD were published; it is interesting that even then, 67–92% of the surveyed ophthalmologists rated genetic counseling to be very important in the prevention of blindness, whereas the doctors in our sample were skeptical about the preventive potential of genetics in AMD.

### Practice implications and research recommendations

Doctors have been envisaged to be key players in properly incorporating progress in genetics and DNA technologies in the health care system. This has been emphasized mainly with a view to hereditary cancer, where doctors are expected to help implement needs-based genetic testing and personalized therapy [37]. In terms of AMD genetics, the results of this present study indicate that many ophthalmologists are neither prepared nor inclined to utilize genetic knowledge in their daily work. Although hundreds of publications on the genetics of AMD have been published in the last decade, the interviewed private practitioners perceived clear knowledge deficiencies and do not feel comfortable with the topic; some even appear not to have come to terms with the concept of multifactorial diseases yet. Ophthalmologists employed by hospitals reported to have better access to genetic information and also benefitted from direct exchange with genetic researchers. The interviews highlight a need for a targeted knowledge transfer which conveys information on AMD genetics to private practitioners in a succinct, understandable way and which gives clear implications for clinical practice. Special trainings and educational interventions that are grounded in the daily practice of ophthalmologists may be useful in informing ophthalmologists about the genetic background of AMD and about appropriate ways to communicate genetic information to patients. In the field of oncogenetics, providing genetic educational outreach was shown to have a moderate effect on physicians’ self-confidence and, in few studies, on reported changes in practice [39–41]. The interventions included short educational sessions, education over longer time spans (e.g. two years), and online educational courses. Prolonged exposure to genetics information (e.g. series of sessions or full-day workshops) tends to be more effective than short or one-off courses [39]. The authors of a recent systematic review on genetic education for primary care conclude that more research is needed in the field, especially on resources and tools (e.g. decision aids, just-in-time-information) that may be required to change medical practice [39].

The overall attitude of the interviewees towards genetics of AMD was so skeptical that even better strategies to distribute and communicate genetics information may be futile, as ophthalmologists may not be willing to invest time in acquiring knowledge and attending educational sessions at all. Knowing about heritability or genetic background of AMD does, for the time being, not influence the treatment of manifest patients, thus the ophthalmologists rated the clinical utility of genetics low. Informing AMD patients that their offspring may carry a certain disease risk was rejected by the majority of interviewees, as was recommending a genetic AMD test to patients with other eye conditions who have relatives suffering from AMD. The main reason was that preventive measures were seen as ineffective, or that the genetic information was considered psychologically unsettling. We found that the focus of ophthalmologists is clearly the management of a manifest disease, and the concept of prevention is not yet well integrated into the routine patient care of the interviewed ophthalmologists. This can also be put down to contradictory or unsatisfying evidence on the effectiveness of different preventive measures (e.g. nutrition), and the unspecific character of preventive lifestyles in question (e.g. not smoking, which could be advised to anyone as it lowers the risk for a multitude of diseases, independent of the genetic risk for AMD).

It has to be discussed whether the ophthalmologic clinic or practice is a suitable place for preventive measures, or whether other channels should be used, e.g. campaigns informing the public about AMD, screening possibilities and risk behaviors. Some doctors also raised the point that it is difficult for them to address accompanying relatives of AMD patients, as those are, strictly speaking, not their patients, and the doctors may even be suspected to just recruit new patients for their practice. This highlights a special need for care concepts for diseases with clear genetic background, as the genetic information has consequences not only for the patient, but also for his or her relative. Practitioners may benefit from guidelines of how to act (or react) without needing to fear that they intrude upon their patient’s and relatives’ privacy or unnecessarily worry them.

On the whole, ophthalmologists may underestimate patients’ interest in prevention and genetics. Studies show that patients would welcome their doctors (e.g. general practitioners) to discuss genetic aspects of their disease with them [38]. Similarly, public attitudes towards genetic testing in Europe are positive: the majority of surveyed individuals or patients, respectively, in different countries agreed with the use of DNA testing for early detection of diseases [42–44]. These studies show that attitudes are usually mixed regarding the consequences of testing, with hopes that their lifestyle and medical care could be adjusted to prevent certain diseases, and concerns that the results could affect their life planning with little clinical benefit. In a very recent study, genetic testing for AMD and an optometrist’s counseling were offered to healthy individuals aged 50–65; the response to the testing procedure and the results was overwhelmingly positive [45]. The views of descendants of AMD patients on genetic testing and potential preventive measures are yet to be explored. If we better understand the needs and fears of those relatives, it will be easier to draft a recommendation for ophthalmologists on how to address accompanying family members of AMD patient.

Many authors have criticized that genomic research discoveries are not translated to be applicable in clinical practice and to population health benefits [46]. In AMD genetics, the gap between genomic research and clinical practice appears to be especially wide, according to the results of the interviews, despite the relatively large genetic risk for this disease. The reason for this is not ignorance or reluctance of ophthalmologists, but rather the lack of translational studies transferring the genomic findings from basic research to clinical research, and from there to evidence-based recommendations for implementation in practice [47]. Anand et al describe that although the number of population-based genetic studies in AMD is increasing every year, most of these findings have not been translated into development of human diagnostic, prognostic and pharmaceutical applications [48]. For example, future studies may investigate whether individuals tested for AMD genes have a lower risk of developing the manifest disease when adhering to a preventive lifestyle, and whether knowing their risk affects their quality of life. This evidence is required in order to inform the patient care of ophthalmologists.

Some authors also point out that translational research and knowledge transfer needs to involve clinicians, proposing that the models conceiving translation as a ‘pipeline’ or a unidirectional pathway (moving from the laboratory to the clinic) need to be overcome in favor of an ‘interlocking loop’ model [49] or a ‘two-way road’ [50]. This view is reverberated in the statements of many interviewees among the private practitioners, who felt that genetic research was conducted in a way that was detached from the realm of patient care, and who called for an interactive communication between ophthalmologists and researchers. In order to feed knowledge from ‘the bedside’ (or the private practice) back into genomic research, new structures for collaborative partnerships need to be developed.

## Conclusion

Genetic research on AMD has made enormous progress over the last decade, showing that several genetic susceptibility factors strongly impact AMD risk. With current evidence of some lifestyle factors modulating epigenetic marks, some of the genetic risk might be modifiable by life style. Our study indicates that this knowledge has not had any impact on clinical ophthalmologic practice yet, neither by private practitioners, nor by ophthalmologists employed by hospitals. Even among those doctors who are aware of the genetic aspects of AMD, many withhold this information from patients and their relatives, because of the uncertainty of predicting AMD and for fear of unsettling those individuals. Preventive efforts for late AMD based on genetic information are seen as irrelevant. These findings highlight a need for genetic educational programs tailored to the concerns and routine care situations of ophthalmologists. With the existing evidence that genetic factors convey a substantial AMD risk, it becomes important to perform studies that involve the relatives of AMD patients and explore their views on information, genetic testing and/or clinical screening. These investigations are fundamental to guide future strategies of ophthalmologists (and, possibly, primary care physicians as well) to address patients whose parents suffer from AMD. In addition, long-term clinical studies need to be initiated to assess the benefit of preventive measures in those individuals that were tested to have an elevated or high genetic risk score for AMD. It is honorable that ophthalmologists intend to act responsibly in the favor of their patients by not unsettling them with uncertain predictions of a disease that may lead to blindness; on the other hand, one has to consider that ‘*undetected genetic risk can have serious consequences for the entire family*, *for example through preventing access to screening or preventive drugs…resulting in increased morbidity…*., *family burden and healthcare costs*’ [39].
